This article has been retracted.

# Analysis of Clinical Related Factors of Severe Mycoplasma pneumoniae Pneumonia in Children Based on Imaging Diagnosis

**DOI:** 10.1155/2022/4852131

**Published:** 2022-02-27

**Authors:** Xiaoshuai Wang, Xiaofei Lin

**Affiliations:** Department of Pediatrics, Huai'an Maternal and Child Health Hospital, Huai'an, Jiangsu, China 223001

## Abstract

Severe pneumonia is a common acute respiratory disease in children, and it has a rapid onset and violent onset, which often affects the whole body. Moreover, typical clinical manifestations and signs often cannot be taken seriously or covered up in clinical work. Due to the short time for treatment, it is easy to cause improper diagnosis and treatment, aggravate the disease and further deteriorate, and even threaten the life of the child. In order to achieve early intervention and treatment of severe Mycoplasma pneumoniae pneumonia in children, reduce or shorten the course of the disease, and improve the cure rate, this paper combines the imaging diagnosis to study the analysis of clinical related factors of severe Mycoplasma pneumoniae pneumonia in children. In addition, this paper analyzes the experimental data with hospital case samples, conducts statistical research on the analysis of clinical related factors of severe Mycoplasma pneumoniae pneumonia in children, and proposes effective coping strategies.

## 1. Introduction

MPP (Mycoplasma pneumoniae pneumonia) is a frequent respiratory ailment in children. In recent years, the risk of Mycoplasma pneumoniae (MP) infection in the Chinese population has increased, and investigations on the epidemiological features of Mycoplasma pneumoniae pneumonia have shown that MPP has an epidemic breakout every 3-4 years in various European countries [1]. Under normal circumstances, MPP is mostly a benign, self-limiting disease. However, drug abuse, drug resistance, clinical misdiagnosis, and missed diagnosis progressively aggravate the disease. The number of children with severe Mycoplasma pneumoniae pneumonia (SMPP) is increasing every year [2]. Therefore, in clinical work, we can identify the clinically relevant factors of SMPP early and intervene and treat them early to reduce or shorten the course of the disease and improve the cure rate.

MP infection is seen in children of all age groups, especially preschool and school-age children, the incidence of MP pneumonia is higher, and its age of onset tends to be younger, and the symptoms vary. Cases of refractory or severe Mycoplasma pneumoniae pneumonia have steadily risen in recent years. This puts the children's health in jeopardy, prolongs their hospital stay, adds to the family's financial load, and may possibly result in catastrophic consequences. The high secretion of airway mucus may be one of its pathogeneses [3]. Mucin generated by airway goblet cells and submucosal glands, as well as water and electrolytes released by airway epithelial cells, make up the majority of airway mucus. It may catch particles and germs as part of the respiratory tract's natural immunological function. Excessive mucus production is a typical clinical feature of airway illnesses such as chronic obstructive pulmonary disease (COPD), bronchial asthma, pulmonary cystic fibrosis, and bronchiectasis, among others. [4]. Thromboxane B2 (TXB2) is a metabolite of arachidonic acid, a key inflammatory mediator that plays a role in a wide range of inflammatory and immunological responses. TXB2 may cause increased vascular permeability in COPD patients, resulting in airway microvascular leakage and increased airway mucus. Smoking-induced increased mucus production may be reduced by blocking the TXB2 receptor.

Severe cases threaten the health and lives of children. Although new antibiotics continue to appear and treatment technologies continue to improve, severe pneumonia is still one of the main causes of death in children under 5 years of age in developing countries, especially in infants and young children, most of which are children. Died from various complications of severe pneumonia. Pediatric pneumonia is a group of respiratory diseases caused by bacteria, viruses, and other causes including foreign bodies. Mild patients can only show general symptoms of pneumonia, such as cough and sputum, fever, and fixed wet rales on lung auscultation, but in recent years, about half of the pediatric intensive care units have had severe pneumonia cases in children. Some patients may continue to develop severe pneumonia due to untimely treatment of mild cases, unreasonable antibiotic application, and self-resistance. In addition to severe respiratory symptoms, some cases may have obvious central nervous system involvement and other systemic symptoms. Community-acquired pneumonia and hospital-acquired severe pneumonia are the two types of severe pneumonia. Acute lung infection with fever, cough, dyspnea, chest depression, pulmonary rales, chest radiographs with infiltrating shadows, etc., is defined as a child who has not been hospitalized in the hospital 14 days before the onset of symptoms and has acute lung infection with fever, cough, dyspnea, chest depression, pulmonary rales, chest radiographs with infiltrating shadows, etc. Acquired pneumonia is pneumonia that does not present at the time of admission and is not in the incubation phase but develops three days after admission or within seven days of discharge. Community-acquired severe pneumonia is the key trend discussed in this article. In the past, severe pneumonia was defined as having associated symptoms and signs affecting the circulatory, neurological, and digestive systems in children with pneumonia. Children with pneumonia are thought to have significant ventilatory dysfunction or inflammatory responses all throughout their bodies. It may be identified as severe pneumonia in the case of severe pneumonia. In children, severe pneumonia is a life-threatening condition caused by a primary lung infection. Intravascular coagulation (DIC), cerebral edema, gastrointestinal dysfunction, and even multiple organ dysfunction syndrome are caused by ventilatory and ventilation disorders, hypoxemia, respiratory failure, acid-base balance, and electrolyte imbalance microcirculation disorder, shock, and even diffusion (MODS). The majority of children in this age range are suffering from severe pneumonia. Different pathogens or other factors (such as inhalation of amniotic fluid, oil, or allergic reactions) cause bronchial mucosal congestion, edema and alveolar congestion, and even release of toxins.

This article combines the analysis of clinical related factors in imaging diagnosis research severe Mycoplasma pneumoniae pneumonia in children to realize early intervention and treatment of patients, reduce or shorten the course of disease, and improve the cure rate.

## 2. Related Work

Humans are generally susceptible to Mycoplasma pneumoniae, and the age characteristics of Mycoplasma pneumoniae infection are clear, that is, it occurs in children over 5 years old. The results of early studies on children with Mycoplasma pneumoniae infection of different age groups and genders are not consistent. Some studies suggest that there are gender differences, but the differences are not very obvious. The gender makeup of the hospitalized patients at the same time is utilized as the backdrop for such studies since the subjects are practically all hospitalized patients. In general, there is no gender difference in Mycoplasma pneumoniae infection in children [5]. Previous research has shown that Mycoplasma pneumoniae infection is uncommon in children under the age of five, with the maximum frequency occurring between the ages of five and fifteen. These investigations are based on serology; however, owing to their impaired immune function, children in the young age range, particularly newborns and young children, have a low positive rate of serological tests, resulting in misleading negative findings [6]. The antibody titers of Mycoplasma pneumoniae in children aged 0 to 3 years were the lowest, while those in children aged 4 to 6 years and more than 7 years were considerably greater [7]. According to the literature [8], infection rates in the 1-2-year-old and 2-3-year-old groups are 32.33 percent and 35.53 percent, respectively, suggesting that Mycoplasma pneumoniae infection in young children is frequent. Reports of Mycoplasma pneumoniae infection in young infants have increasingly grown as detection technology has improved, particularly with the introduction of the molecular biology technique PCR. The literature [9] used real-time PCR to detect the P1 gene of Mycoplasma pneumoniae in throat swabs and found that 12% (102/886) of children had a positive PCR test result. Among them, 22.57% of the positive children are younger than 2 years old, which is lower than the positive detection rate of 41.2% in the 5-9-year-old group, but slightly higher than the positive detection rate of 20.6% in the 10-14-year-old group. Molecular epidemiological studies in Suzhou area indicate that Mycoplasma pneumoniae infection is also common in young children. Among them, the proportion of the July 1-year-old group is 19.46%, and the proportion of the 13-month-old group is 33.0%.

Mycoplasma pneumoniae infection may induce not only upper respiratory tract infection but also lower respiratory tract infection, whether in an epidemic or nonepidemic era. Pneumonia is a severe complication of a respiratory illness. Parts of the symptoms of Mycoplasma pneumoniae infection in children might last for weeks or months. As a result, infection with Mycoplasma pneumoniae is one of the most common causes of persistent cough and recurrent respiratory infections [10]. Drug-resistant Mycoplasma pneumoniae strains have been regularly documented, and refractory and severe Mycoplasma pneumonia has steadily grown in recent years, notably in Asia, which may be associated with Mycoplasma pneumoniae macrolide antibiotic resistance [11]. The frequency of macrolide-resistant Mycoplasma pneumoniae was researched in the literature [12], and the 5-year drug resistance rates were 68.9%, 90.0 percent, 98.4 percent, 95.4 percent, and 97.0 percent, respectively. In recent years, the link between Mycoplasma pneumoniae infection and asthma has gotten a lot of attention. Mycoplasma pneumoniae might have a key role in the onset, progression, and chronicity of asthma [13]. Except for respiratory diseases, extrapulmonary complications caused by Mycoplasma pneumoniae infection have gradually attracted people's attention. The mechanism of Mycoplasma pneumoniae infection and involvement of the external organs of the lung is not fully understood. Some people think that because Mycoplasma pneumoniae antigens and the human heart, liver, lung, brain, kidney, and smooth muscle tissues have some common antigens, they can be produced when Mycoplasma pneumoniae is infected. Corresponding autoantibodies and the formation of immune complexes cause disease in other target organs outside the respiratory tract, and the appearance of the corresponding extrapulmonary system involvement [14]. It usually occurs within 7-14 days of the disease, and most of them are older children. Common extrapulmonary complications include damage to the nervous system, cardiovascular system, urinary system, blood system, digestive system, and skin, and occasionally, arthritis, Kawasaki disease, papilledema, and iritis have been reported [15].

Clinically, mixed infection of Mycoplasma pneumoniae pneumonia is not uncommon. The mixed virus infection rate of Mycoplasma pneumoniae infection in children investigated in the literature [16] was 14.5%; the most common was combined respiratory syncytial virus infection, followed by human bocavirus and parainfluenza virus 3. Literature [17] found that among children under 5 years of age with acute respiratory infections, the mixed infection rate of Mycoplasma pneumoniae was 19.3%. Different detection pathogen spectrums will lead to inconsistent final results. Therefore, a large sample multicenter study with the same methodology is still needed to confirm [18].

Mycoplasma pneumoniae, like Streptococcus pneumoniae, Staphylococcus aureus, and other bacteria, has a colonization state, also known as a carrier state. Mycoplasma pneumoniae can survive in the respiratory tract for several months or even longer after infecting the body, mainly because Mycoplasma pneumoniae can firmly adhere to the airway epithelial cells after infecting the body, and even invade the airway epithelial cells, forming asymptomatic pneumonia. The condition of recessive infection is also known as colonization or carrier status [19]. Mycoplasma pneumoniae infection may be passed down through the generations; however, most cases are asymptomatic and recessive [20]. Clinicians need to know how to tell the difference between infection and colonization state. They can identify the pathogen and ensure that antibiotics are used appropriately, while also avoiding antibiotic overuse and the development of drug-resistant strains. This difficulty might be solved by using quantitative PCR to detect the load of Mycoplasma pneumoniae. Serum IgM positivity is much lower in children with low mycoplasma pneumonia load than in children with high load, and mixed infections are uncommon in children with high load [21]; at the same time, mycoplasma in the alveolar lavage fluid of children with refractory mycoplasma pneumonia. The load is significantly higher than that of nonrefractory children [22], all of which indicate that low load may be a colonization state to a certain extent, but it needs to be confirmed by advanced studies.

## 3. Materials and Methods

We collected hospital-treated children with Mycoplasma pneumoniae pneumonia in children as the observation group and 30 normal children who had a physical examination in the hospital during the same period as the control group. Moreover, we retrospectively analyzed the clinical data of the two groups to explore the related risk factors of severe Mycoplasma pneumoniae pneumonia in children.

All selected children with severe pneumonia conform to the WHO concept of severe pneumonia in the prevention and treatment of acute respiratory infections in children: lethargy or agitation, refusal to eat, depression of the lower chest wall, and cyanosis. Diagnostic criteria: ① the patient has significant symptoms of nervous system poisoning: lethargy, prolonged awakeness, poor spirits, repeated cramps, etc.; ② the patient has significant dyspnea and hypoxia, and the symptoms cannot be relieved after oxygen inhalation; ③ the patient has circulatory system manifested as heart failure; ④ the patient's physical signs shows wet rales on lung auscultation, bronchial breath sounds, dullness on percussion, and diffuse shadows on imaging examination; ⑤ the patient has very serious complications: such as empyema, sepsis, and toxic encephalopathy. Those with more than one of the above diagnostic criteria are diagnosed with severe pneumonia. However, those without the above diagnostic criteria are diagnosed as ordinary pneumonia.

We retrospectively analyzed the clinical manifestations and signs, underlying diseases, pathogenic examinations, and imaging of hospitalized children with severe pneumonia (observation group) and compared them with those of ordinary pneumonia hospitalized in the same period (control group).

## 4. Result

All children in the observation group have fever. Among them, 50.8% of children have a body temperature of 39°C-41°C, 75% of children have a heat duration of more than 7 days, 94.8% of children have a cough, and 58.5% of children have a respite. All children have dyspnea, shortness of breath, or cyanosis, and 14.1% of them required mechanical ventilation. The children with wet rales account for 54.3%. There are 58.5% of children with underlying diseases, including 29% of congenital heart disease, 21.2% of malnutrition, and 8.3% of other diseases. Children with respiratory failure account for 78.7%, children with acute respiratory distress syndrome account for 6.2%, children with heart failure account for 84.5%, and children with abdominal distension account for 34.7%. Children with common pneumonia in the control group all had fever. Among them, 34.2% of children have a body temperature of 39°C-41°C, 92.5% have a heat duration of less than 7 days, 63.3% have a respite, and 19.2% of children have a respite have dyspnea. Children with underlying diseases accounted for 20.8%, including congenital heart disease and malnutrition. The detailed comparison is shown in Table 1 and Figure 1. There was no significant difference in the composition ratio of the clinical manifestations of cough and wheezing between the two groups of children (*P* > 0.05). However, there is a statistically significant difference between the two groups of children in high fever (body temperature between 39°C and 41°C), heat duration greater than 7 days, dyspnea, shortness of breath or cyanosis, dry or wet rales in the lungs, and underlying diseases (*P* < 0.05). Severe pneumonia and common pneumonia basically have cough and wheezing. However, if the child has fever for a long time, high fever, dyspnea, shortness of breath, or clinical manifestations of cyanosis, and positive lung signs, accompanied by underlying diseases, beware of the possibility of severe pneumonia. This is of great significance for our early identification of severe pneumonia.

In the observation group, 47.2% of patients with severe pneumonia-specific Mycoplasma pneumonia antibody (MP-IgM) are positive. When the respiratory virus antibody test is performed, 10.4% of the positive antibodies are detected. When using body fluid culture (sputum culture, pleural fluid culture, and blood culture), 16.1% of positive strains are cultured. Among them, Pseudomonas aeruginosa is 3.6%, Escherichia coli is 3.1%, Klebsiella pneumoniae is 3.1%, Bacillus cloacae is 2.6%, Streptococcus pneumoniae is 1.6%, Streptococcus viridans is 1.0%, Staphylococcus haemolyticus is 0.5%, Agrobacterium radiobacter is 0.5%, and the fungus is Candida, and the ratio is 1.0%. The positive rate of serum-specific Mycoplasma pneumoniae antibody (MP-IgM) in the control group is 26.7%, and the positive antibody detected by the respiratory virus antibody test is 14.2%. Compared with the observation group, there is a difference (*P* < 0.05), and most of the children with severe pneumonia were infected by bacteria or mycoplasma. See Table 2 and Figure 2 for specific comparison.

Imaging examinations were performed on 193 children with severe pneumonia in the observation group. The child showed pulmonary lobes or segmental large patches of increased density or inflammatory and infiltrating lung parenchymal lesions. Among them, 54.9% of children meet the diagnostic criteria for lobar pneumonia, and 33.2% of children meet the pulmonary interstitial inflammatory lesions (such as increased lung texture, blurring, and flocculation of inner and middle bands), 15.5% of children meet the pleural effusion, 8.3% of children meet the empyema, and 9.3% of children meet the atelectasis. In the control group, 7.5% of the children meet with lobar pneumonia, 77.5% of the children meet with interstitial pneumonia, 4.2% of the children meet with pleural effusion, and 2.5% of the children meet with atelectasis. The specific comparison is shown in Table 3 and Figure 3. It can be seen that children with severe pneumonia are mainly characterized by lobar pneumonia, and children with common pneumonia are mainly characterized by lobular pneumonia (interstitial changes). Therefore, imaging examination is helpful for the early diagnosis of severe pneumonia and is very important for the prognosis of children.

Oxygen, nebulized sputum suction, ECG monitoring, and complete therapy are all frequently provided to patients. Controlling inflammation, improving ventilation, treating symptoms symptomatically, and preventing and treating complications are the guiding concepts. We must pay close attention to water and electrolyte supplementation, as well as the correction of acidosis and electrolyte abnormalities. Patients are given anti-infective and antiviral therapies based on their history or pathologic outcomes. Empirical antibiotics, for example, do not improve their health, and antibiotics are modified over time depending on drug sensitivity data or potential infections to expand pathogen coverage. Parenteral antibiotic therapy, particularly intravenous antibiotic therapy, is the first line of treatment for severe pneumonia. The idea is to choose sensitive medications depending on germs that cause disease. To guide therapy, suitable respiratory secretions should be obtained for bacterial culture and drug sensitivity testing before taking antibiotics. You might pick sensitive medications based on experience before acquiring the culture results. The selected drugs should have a higher concentration in the lung tissue, early medication, combined medication, sufficient amount, and full course of treatment. Antibiotic therapy and prognosis for severe pneumonia normally last 5-7 days after the body temperature returns to normal, and the medicine is terminated three days after the symptoms, and signs have gone away. The body's susceptibility to medications should be taken into account, and the condition and effectiveness of the therapy should be assessed 48 hours after it begins. Patients should be considered ineffectual if their symptoms do not improve or worsen after 72 hours of first therapy, and antibacterial medicines should be carefully adjusted. Antibiotics need to be selected according to different pathogens, penicillin is the first choice for Streptococcus pneumoniae, and macrolide antibiotics such as erythromycin should be used for those who are allergic to penicillin. Cloxacillin sodium is the first choice for Staphylococcus aureus, and vancomycin or combined with rifampicin is used for resistant patients. Amoxicillin and clavulanic acid are preferred for Haemophilus influenzae, ceftriaxone is preferred for Escherichia coli and pneumoniae, and ticarcillin and clavulanic acid are preferred for Pseudomonas aeruginosa. Patients with liver function and myocardial damage are given liver-protecting and heart-protecting treatments, and nutritional support treatment is strengthened at the same time. The application period of intravenous gamma globules is generally in severe infections and severe systemic inflammation, which effectively controls the development of the disease and promotes the recovery of the disease. In addition, patients with pneumothorax, mediastinal emphysema, and empyema need to be treated with closed thoracic drainage and mediastinal exhaust. Finally, patients with dyspnea and hypoxemia need to adopt the priority strategy of CPAP, and those who meet the indications for the computer are given tracheal intubation and mechanical ventilation.

## 5. Analysis and Discussion

Ambulatory infiltration is sometimes a thin cloud-like infiltration shadow. Therefore, for further understanding of severe pneumonia, it is necessary to pay close attention to the chest X-ray examination. X-ray is the objective evidence for judging pneumonia, and its manifestations may have flaky shadows or changes in lung texture. At the same time, it can also help you distinguish between bronchial pneumonia and lobar pneumonia in the clinic, and it has a certain prompting effect on bacterial or viral and mycoplasma infections. It may also aid in the treatment of TB, lung cysts, bronchial foreign bodies, and other disorders that cause shortness of breath and death. As a result, imaging studies must be included in clinical practice in order to detect critically unwell children early. Severe pneumonia in children is a dangerous condition that pediatricians devote special attention to. Severe respiratory depression and partial involvement of the brain neurological system may hasten the progression of the illness, resulting in severe empyema, systemic infection, and possibly shock. The preservation of normal respiratory function is especially important as a result of comprehensive therapy that includes phlegm, anti-infection, or antivirus. Pathological alterations such as increased airway secretions, microvascular spasm, and airway stenosis are common in severe pneumonia. At the same time, the normal clearance of cilia decreases and the physiological barrier function decreases, all of which promote the occurrence and development of pneumonia to a certain extent. For some patients with severe pneumonia combined with significant decline in immune response and prodromal hypotension, the therapeutic effect of oxygen inhalation through the nasal cannula is not obvious. Moreover, mechanical ventilation poses the risk of damage to the mucous membrane of the respiratory tract. In addition, delayed lung ventilation and poor ventilation function caused by ventilator-associated pneumonia limit its application in patients with severe pneumonia. In recent years, the maintenance of positive end-respiratory pressure and continuous ventilation can significantly improve children's exhalation and inspiratory dysfunction.

## 6. Conclusion

Clinical pediatricians should have a full understanding of the diagnosis of severe pneumonia. The pathogenesis of severe pneumonia in children is quite different from that of ordinary pneumonia, and severe pneumonia has a greater impact on the life safety of children. The onset of severe pneumonia is more rapid, and clinicians can make accurate judgments on the symptoms and signs of the onset. Children with severe pneumonia generally present with cough, wheezing, high fever, fast heart rate, etc. There are obvious wet rales in the lungs. These manifestations are a greater threat to the health of the children. However, there is also severe pneumonia with fever and cough in the early stage, and the lung signs have no obvious specificity. They are often difficult to distinguish from other respiratory tract infectious diseases that are onset in infants and young children and can easily be misdiagnosed. With the progress of the disease, due to the persistent high fever, the large-lobe consolidation of the lungs in imaging studies and the ineffectiveness of antibiotic treatment have attracted attention. At this time, the lung damage is aggravated, and the lung consolidation is accompanied by pleural effusion and empyema on the basis of imaging. The emergence of multiple system complications makes the treatment more difficult, and the prognosis is poor. Moreover, the early and effective application of antibiotics is particularly important for the prognosis of severe pneumonia, while supportive treatment also plays an important role. The enhancement of children's immunity and vaccination also play a certain role in the prevention of pneumonia.

## Figures and Tables

**Figure 1:** Statistics on comparison between severe pneumonia and common pneumonia.

**Figure 2:** Statistical diagram of comparison of the etiology of severe pneumonia and common pneumonia.

**Figure 3:** Statistical diagram of comparison of analysis of imaging of severe pneumonia and common pneumonia.

**Table 1:** Comparative analysis of severe pneumonia and common pneumonia.

Group	High fever	Heat course is greater than 7 days	Cough	Respite	Difficulty breathing, rales in the lungs	Shortness of breath, cyanosis	Basic illness
Observation group	50.78%	42.49%	94.82%	58.55%	100.00%	54.40%	58.55%
Control group	34.17%	0.00%	92.50%	63.33%	19.17%	70.83%	20.83%
*χ* ^2^	8.3527	—	0.70498	0.71508	—	8.45673	43.12599
*P*	<0.05	<0.01	>0.05	>0.05	<0.01	<0.01	<0.01

**Table 2:** Comparison of the etiology of severe pneumonia and common pneumonia.

Group	Observation group	Control group	*χ* ^2^	*P*
Germ	16.06%	6.67%	5.846	<0.05
Virus	10.36%	14.17%	1.037	>0.05
Mycoplasma	47.15%	26.67%	13.145	<0.01

**Table 3:** Comparison of analysis of imaging of severe pneumonia and common pneumonia.

Group	Lobar pneumonia	Interstitial pneumonia	Pleural effusion	Atelectasis	Empyema
Observation group	54.92%	33.16%	15.54%	9.33%	8.29%
Control group	7.50%	77.50%	4.17%	2.50%	0.00%
*χ* ^2^	72.311	58.771	8.617	4.517	—
*P*	<0.01	<0.01	<0.05	<0.05	<0.01

## Data Availability

The data used to support the findings of this study are included within the article.
